# A Rare Case of Gemella haemolysans Endocarditis: A Challenging Diagnosis

**DOI:** 10.7759/cureus.52030

**Published:** 2024-01-10

**Authors:** Nadine S Kassab, Noor Alsammarraie, Tania Sarsam, Mina Al-Sammarraie, John Watt

**Affiliations:** 1 Internal Medicine, Trinity Health Ann Arbor Hospital, Ypsilanti, USA; 2 Otolaryngology, Royal Sussex County Hospital, Brighton and Hove, GBR; 3 Internal Medicine, Ibn Al Haytham Hospital, Amman, JOR

**Keywords:** beta lactam antibiotics, septic brain embolism, bacterial sepsis, valve vegetation, gemella endocarditis

## Abstract

*Gemella haemolysans* bacterium is an opportunistic pathogen that can cause localized or systemic infections. Here we describe a rare case of infective endocarditis secondary to *Gemella haemolysans* infection. In our case, although the bacteremia was cleared with antibiotics, the mitral valve vegetations continued to enlarge and the course was complicated by septic brain emboli.

## Introduction

*Gemella* is a gram-positive, catalase-negative, facultative anaerobic coccus. It is part of the normal flora that colonizes the human mucous membranes, including the oropharynx, the genitourinary, and the gastrointestinal tract. It can cause local and systemic infections such as osteomyelitis, endocarditis, and central nervous system (CNS) infections [1-12]. *Gemella* endocarditis most commonly affects the mitral and aortic valves. *Gemella* is highly susceptible to β-lactams; however, in resistant cases, vancomycin can also be used [11-13]. Here, we present a case of *Gemella haemolysans* endocarditis involving a native mitral valve complicated by septic emboli to the brain.

## Case presentation

A 77-year-old female with end-stage renal disease (ESRD) on peritoneal dialysis, paroxysmal atrial fibrillation, hypertension, hyperlipidemia, and diabetes mellitus on insulin, was admitted with a two-week history of malaise, dizziness, and poor appetite. She also had a few days’ history of left shoulder pain following a recent shoulder injury. On admission, she had a temperature of 38.2° C, a heart rate of 108 bpm, and a blood pressure of 96/64 mmHg. She was alert and oriented without a focal neurological deficit. She had normal breath sounds and a systolic murmur on auscultation. Her left shoulder was tender to palpation with a reduced range of movement, without erythema or swelling. Laboratory values were significant for WBC of 28.8 K/uL. Urinalysis was positive for leukocytes but negative for nitrites. Chest x-ray showed cardiomegaly unchanged from previous imaging (Figure 1). CT head, chest, abdomen, and pelvis showed no acute abnormalities. A left shoulder x-ray showed a possible small effusion (Figure 2). Urine culture grew *Escherichia coli*.

**Figure 1:** Chest x-ray showing cardiomegaly

**Figure 2:** Shoulder x-ray showing a possible small effusion

The patient was treated empirically with IV cefepime and vancomycin. On day 3 of hospitalization, the patient became agitated and confused. There was no nuchal rigidity on examination. By day 4, *Gemella haemolysans* bacteremia grew in 4/4 of blood cultures. Therefore, vancomycin and cefepime were switched to IV ceftriaxone 2g daily as *Gemella* is highly susceptible to β-lactams. In an attempt to localize the primary source of infection, the literature was searched for the most common sources of infection with this bacterium. It was found that *Gemella* can cause endocarditis, osteomyelitis, and CNS infections. Given the patient’s complaints of left shoulder pain, and the finding of shoulder x-ray suggestive of joint effusion, synovial fluid aspiration was performed for cell count, culture, and sensitivity, which were negative. The peritoneal fluid culture was negative. Endocarditis was also suspected in the setting of sepsis, new murmur, and new encephalopathy. Therefore, a transthoracic echocardiogram (TTE) was performed showing mildly thickened mitral valve leaflets with trace mitral regurgitation. Transesophageal echocardiogram (TEE) showed large mobile vegetation on the anterior leaflet of the mitral valve of 1.3 cm (Figure 3). Given the patient's new encephalopathy in setting off endocarditis, a brain MRI was performed showing septic emboli with acute infarcts throughout the cerebral and cerebellar hemispheres (Figure 4). On further questioning for the site of pathogen entry, the patient's family denied any recent dental procedures or colonoscopies. Maxillofacial surgery evaluation for a possible dental source was negative for dental abscesses.

**Figure 3:** Transesophageal echocardiogram showing a large mobile vegetation (1.3 cm) on the anterior leaflet of the mitral valve

**Figure 4:** Brain MRI showing multiple infarcts throughout the cerebral hemispheres suggestive of septic emboli

Despite being on antibiotics, the patient did not have any clinical improvement. Blood cultures were repeated without microorganisms' growth. IV ceftriaxone was continued. Additionally, the patient was deemed a non-surgical candidate on cardiothoracic surgery evaluation. A week later, the patient's encephalopathy worsened, and she was only responsive to painful stimuli. EEG showed diffuse encephalopathy. A repeat MRI of the brain showed multiple new punctate foci suggestive of acute embolic infarction. TEE was repeated showing enlargement of vegetation to 2.1 cm (Figure 5). Recovery without source control seemed unlikely. The case was discussed with multidisciplinary teams at multiple quaternary medical centers who also deemed the patient not a surgical candidate due to her multiple comorbidities and progressive debility. Considering her poor prognosis, the patient was transitioned to comfort measures and passed away a few days later.

**Figure 5:** Transesophageal echocardiogram showing enlargement of the vegetation (2.1 cm) on the anterior leaflet of the mitral valve

## Discussion

*Gemella* species are part of the normal flora of the human mucus membranes. *Gemella haemolysans* is an opportunistic organism that can cause infections such as meningitis, osteomyelitis, septic shock, and, rarely, as in our reported case, infective endocarditis. It is reported that *Gemella* accounts for less than 1% of endocarditis cases. Sixty-six cases of *Gemelli*-associated endocarditis were reported in the literature up until 2019 [1-8]. It can cause life-threatening infections in patients with predisposing risk factors, such as advanced age, with a mean age of 50 [1-7]. The most commonly known source is dental infections from poor dental hygiene and manipulation. Other sources include gastrointestinal procedures such as colonoscopies, colon malignancies, preexisting cardiac pathologies, IV drug use, steroid therapy, and diabetes mellitus [2,3,5,7]. Our case illustrates atypical findings with predisposing risk factors including peritoneal dialysis, diabetes mellitus, and advanced age. Similar to our case, onset is usually subacute, and the mitral valve is the most affected.

Most of the cases that were successfully treated with antimicrobial therapy alone, were susceptible to β-lactam antibiotics, especially ceftriaxone, as well as penicillin in combination with aminoglycosides. In penicillin-allergic or resistant cases, vancomycin monotherapy or erythromycin plus rifampicin combination was used [11]. Half of the cases with affected cardiac valves required surgical valve replacement, especially cases with large vegetations, antibiotic-resistant infections, or progressive heart failure [6-9]. In our case, subsequent blood cultures were negative following antibiotics use but the vegetation continued to enlarge despite two to three weeks of IV ceftriaxone which was believed due to the inability of the antibiotics to penetrate the large vegetation. As a result, our patient continued to have septic emboli in the brain. Surgical treatment was indicated in our case with the occurrence of septic emboli and large vegetation not responding to antibiotics alone, but unfortunately, due to multiple comorbidities, she was not deemed a surgical candidate.

Literature search showed that *Gemella* endocarditis is associated with an overall mortality in 18% of the cases, with no significant difference between those who received medical management alone versus those who underwent surgery [1]. Our case demonstrated the challenge and seriousness of diagnosing and managing *Gemella* endocarditis, which adds to the literature to heighten physicians’ awareness and knowledge about a microorganism that can cause significant morbidity and mortality with delayed diagnosis and treatment.

## Conclusions

*Gemella* endocarditis is an unusual and potentially fatal infection that has a tendency to develop large vegetations causing septic brain emboli. The diagnosis is usually challenging and delayed as blood cultures can take up to four days to grow, as in our case. We report this case to heighten physicians' awareness of this rare bacterium as a cause of infective endocarditis. Although bacteremia clearance can be achieved with β-lactam antibiotics, in half of the cases antibiotics therapy alone may not be sufficient to penetrate the large vegetation, and surgical intervention may therefore be warranted.
